RETRACTED

# Application of Graph Neural Network in Driving Fatigue Detection Based on EEG Signals

**DOI:** 10.1155/2022/9775784

**Published:** 2022-08-23

**Authors:** Zhendong Mu, Ling Jin, Jinghai Yin, Qingjun Wang

**Affiliations:** ^1^The Center of Collaboration and Innovation, Jiangxi University of Technology, Nanchang 330098, Jiangxi, China; ^2^College of Economics and Management, Shenyang Aerospace University, Shenyang 110136, Liaoning, China; ^3^Nanjing University of Aeronautics and Astronautics, Nanjing 210016, China

## Abstract

The objective of this article is to solve the current social phenomenon of a large number of fatigue driving, so that social safety becomes more stable in the future, and the detection and application of driving fatigue are more meaningful. This article aims to study the application of graph neural network (GNN) in driving fatigue detection (this article is abbreviated as DFD) based on EEG signals. This article uses a pattern classification method based on a multilayer perceptual overlimit learning machine to find the hidden information of the signal through an unsupervised learning self-encoding structure, which achieves the optimization purpose and has a better classification effect than traditional classifiers. An improved soft threshold (the soft threshold can be used to solve the optimization problem, and the optimization problem solved is similar to the base pursuit noise reduction problem, but it is not the same, and it should be noted that the soft threshold cannot solve the base pursuit noise reduction problem) denoising algorithm is selected, and the collected EEG (a technique for capturing brain activity using electrophysiological markers is the electroencephalogram). The sum of the postsynaptic potentials produced simultaneously by a large number of neurons occurs when the brain is active. It records the process of brain activity in the cerebral cortex or scalp surface) signals are preprocessed, so that the feature extraction efficiency of extracting EEG signals is improved. The final experimental data show that the traditional support vector machine, SVM algorithm, and the KNN convolutional neural (the K-nearest neighbor method, often known as KNN, was first put forth by Cover and Hart in 1968. It is one of the most straightforward machine learning algorithms and a theoretically sound approach) algorithms has a recognition rate of 79% and 81% for fatigue. The improved algorithm in this article has an average recognition rate of 87.5% for driver fatigue, which is greatly improved.

## 1. Introduction

With the rapid development of industrial technology, automobiles have become one of the important tools for transportation; vehicles such as bicycles, cars, motorcycles, trains, ships, and aircraft are commonly used. According to the news released by the Traffic Management Bureau of the Ministry of Public Security in early 2017, as of the end of 2016, the number of cars registered by the Traffic Management Bureau has reached 194 million, and the number of car drivers has exceeded 310 million. The average number of private cars per 100 households in the country has reached. There are 36 vehicles, many of which have more than 70 private cars per 100 households in first- and second-tier cities. There is no doubt that the number of motor vehicles and drivers has increased rapidly, indicating that motor vehicles have become one of the most important modes of transportation in modern China, and the popularity of motor vehicles has brought convenience to people's production and life. These “steel torrents” will also bring some safety hazards to highway traffic. The long working hours of laborers lead to their mental fatigue, thereby increasing the probability of traffic accidents.

RETRACTED

In recent years, with the rapid development of industrial technology, automobiles have become one of the important means of transportation. At the same time, traffic accidents caused by fatigue driving are also increasing year by year. Therefore, how to spot a driver who is fatigued has recently become a hot topic. Previously, most of the research on DFD was based on the recognition of behavioral features and facial expression image features, and the development of brain-computer interface systems has also made it possible to evaluate mental fatigue through EEG signals, which has contributed to driving fatigue based on EEG signals. Related research: due to the high cost of acquisition equipment and inconvenience to wear, fatigue detection based on EEG signals still cannot be applied to civilian use, and it is still in the research stage. However, in recent years, with the development of EEG collection technology and wireless communication technology, brain-computer interface devices have begun to develop, and many portable commercial brain-electricity acquisition devices have gradually appeared on the market. These portable the development of EEG acquisition equipment has greatly reduced the requirements and limitations of EEG acquisition equipment for drivers, and has promoted the development of DFD based on EEG signals.

Research on EEG signals has not stopped all over the world, and various scholars have their own views on this. The following are the results of the research on EEG signals. Liu et al. proposed a method that uses discrete wavelet transform and metaheuristic optimization threshold to automatically remove blinking artifacts from damaged EEG signals. Two metaheuristic algorithms, particle swarm optimization and gray wolf optimization, are used to optimize AC thresholds of different levels for comparison. Although the method they proposed can automatically remove blinking artifacts, it is not very suitable for feature extraction of EEG signals [1]. To better understand false memory, Li and Zheng enhanced the Deese–Roediger–McDermott paradigm experiment. The major causes of the difference in the occurrence of false recollections between the two groups may be discovered to be the participants' emotional states and the brains' comprehension of semantics. Although their improved method can study false memory, there is still a long way to go before such research is applied in real life [2]. Cheng et al. use the learning process to decode EEG signals and establish a recognition mechanism to recognize movement intentions in brain-computer interaction and enable the device to predict human behavior and react in advance. Their research has further deepened the understanding of the relationship between central nervous system signals and hand movements. Although their method can recognize movement intentions in brain-computer interaction, it is based on the premise of upper limb movement intention recognition and cannot be really applied in real life [3]. Although these research methods promote theoretical research to some extent, they have few practical applications and little practicability, so the method proposed in this article has great research significance and value after practical testing.

RETRACTED

The innovations of this article are as follows: (1) a pattern classification method based on multilayer perceptual overlimit learning machine is implemented: H-ELM can search for hidden information of the signal through an unsupervised learning self-encoding structure. The experiment compares PSO-feature classification results of the H-ELM method, H-ELM, and traditional methods to verify that the new method not only achieves the optimization purpose, but also has a better classification effect than traditional classifiers. (2) The improved soft threshold denoising algorithm with the best denoising effect is selected. First, the generation mechanism, characteristics, and classification of EEG signals are introduced, and common EEG signal analysis methods are introduced. Then, a simulation driving EEG signal acquisition experiment is designed and the collected EEG signals are preprocessed.

## 2. Application Method of  GNN  in DFD Based on EEG Signals

### 2.1. Generation Mechanism of EEG Signals

The brain is the most complicated and mysterious organ in the human body, and there are many mysteries that have not been completely solved yet. For example, how the human brain is constructed and how the work between the nerves of the human brain works so well [4]. Generally speaking, the brain includes the three main components of the cerebrum, cerebellum, and brain stem [5]. Among them, the brain has the largest volume and is the high-level nerve center responsible for human thinking activities [6].

RETRACTED

The structure of the EEG signal is shown in Figure 1.

As shown in Figure 1, it is a structure diagram of nerve cells. By querying the data, it can be found that action potentials will be generated after stimulating the dendrites of nerve cells [7]. EEG signals are made up of electrical signals produced by a large number of nerve cells in the brain [8].

### 2.2. GNN Training

The World Wide Web, protein interaction networks, social networks, knowledge graphs, as well as other major real data sets all exist as graphs or networks [9, 10]. However, until recently, few people have paid attention to and studied the use of general neural network models to process data sets of this structure [11]. In the past few years, some articles have reconsidered how to use a universal network to deal with the problem of arbitrary graph structure data, and some of them have achieved excellent results in some fields. The method is dominated by the method based on graph regularization and other methods [12]. How to adapt the neural network model has been studied a lot, such as recurrent neural network (recurrent neural network belongs to deep learning algorithm, its hierarchical structure is tree-like, and the input information is carried out according to the connection order of network nodes) or convolutional neural network, and for any graph, structure is a very challenging problem. Some recent articles introduce network architectures for specific problems, and other articles use the known graph convolution process in the theory of spectral methods to define parameterized filters and apply them to multilayer neural network models [13]. Recent related work has focused on reducing the gap between the fast heuristic learning approach (the heuristic algorithm is used relative to the optimization algorithm. Heuristic algorithm is an intuition-based or experienced algorithm that can search for the best solution within the acceptable computational cost, such as computing time, and occupied space, but does not guarantee finding a feasible or optimal solution; in most cases, the approximation of the optimal solution cannot be explained) and the slow but following certain principles or spectral methods [14].

As shown in Figure 2, the GNN model uses Chebyshev polynomials (the Chebyshev polynomial is an important special function named after the famous Russian mathematician Chebyshev. It originates from the expansion of the cosine function and the sine function of multiple angles; it is related to De Mevre's theorem and is defined recursively; polynomial sequences are a special class of functions in computational mathematics) and some free parameters learned by neural network models to approximate the smoothing filter in the spectral method, and have achieved convincing results in the conventional field [15, 16]. The result is very close to the simple 2D convolutional neural network model [17]. A similar approach is adopted for the graph convolution based on the spectral method, and then a simplified graph convolutional neural network model with significantly faster training time and higher accuracy is introduced, and it has achieved a high level on many benchmark data sets [18].

RETRACTED

In recent years, most GNN models have a certain degree of commonality in architecture and structure. These models can be collectively called graph convolutional networks (GCNs) [19].

### 2.3. Support Vector Machine

For the two types of linearly separable samples, suppose the training sample is {(*y*_*j*_, *x*_*j*_), *j*=1,2,…, *n*}, where *y*_*j*_ is the sample feature vector and *n* is the sample score, then all sample classifications need to meet the following constraints:

(1) $$\begin{array}{c} x_{j}.\left(\varpi .y_{j}+a\right)\geq 1,\;j=1,2,\ldots ,n. \end{array}$$

Among them, the mathematical expression of the hyperplane is as follows:

(2) $$\begin{array}{c} \varpi .y+a=0. \end{array}$$

The distance between the optimal plane to be searched by the support vector and the classification plane is as follows [20]:

(3) $$\begin{array}{c} d=\frac{f\left(y\right)}{\left\|\varpi \right\|}=\frac{1}{\left\|\varpi \right\|}. \end{array}$$

At this time, if the maximum value of the distance (2/‖*ϖ*‖) is required, the problem becomes the minimum value problem.

The Lagrange function (the Lagrangian function, which describes the dynamic state of the entire physical system, is a function that solely incorporates conservative forces in the mechanical system) expression is introduced as follows [21]:

(4) $$\begin{array}{c} L\left(\varpi ,a,\alpha \right)=\frac{1}{2}{\left\|\varpi \right\|}^{2}-\sum_{j=1}^{n}\alpha_{j}\left[x_{j}.\left(\varpi .y_{j}+a\right)-1\right]. \end{array}$$

The partial derivative of the weight vector *ϖ* and the bias a in the above formula can be found, as long as the partial derivative is 0 at the saddle point of the function. At this time, the optimal classification surface problem is transformed into a dual problem, the formula is as follows:

(5) $$\begin{array}{c} \max Q\left(\alpha \right)=\sum_{j=1}^{n}\alpha_{j}-\frac{1}{2}\sum_{j,i=1}^{n}\alpha_{j}\alpha_{i}x_{j}x_{i}\left(y_{j}.y_{i}\right),\\ \text{s.t. }\sum_{j=1}^{n}\alpha_{j}x_{j}=0,\\ \;\alpha_{j}\geq 0. \end{array}$$

The following is available:

(6) $$\begin{array}{c} \varpi^{*}=\sum_{j=1}^{n}x_{j}\alpha_{j}^{*}y_{j}. \end{array}$$

The optimal weight vector and optimal bias must satisfy the following:

(7) $$\begin{array}{c} \alpha_{j}^{*}\left[x_{j}.\left(\varpi^{*}.y_{j}+a^{*}\right)-1\right]=0,\;j=1,2,\ldots ,n, \end{array}$$

and then get the final classification function as follows:

(8) $$\begin{array}{c} f\left(y\right)=\mathrm{sgn}\left\{\left(\varpi^{*}.y+a^{*}\right)\right\}=\mathrm{sgn}\left\{\sum_{j=1}^{n}\beta_{j}^{*}x_{j}\left(y_{j}.y\right)+a^{*}\right\}. \end{array}$$

In reality, linear signals only account for a small part of all signals, and most of the signals that need to be processed are nonlinear signals. For these nonlinear signals, the classification effect of linear support vector machines is not ideal, and support is needed at this time. The vector machine finds a method in the feature space to effectively classify the two types of signals [22, 23].

RETRACTED

Assuming that the initial feature space is *z*, the mapping from the input space to the new feature space is as follows:

(9) $$\begin{array}{c} \varphi \left(z\right)={\left(\varphi_{1}\left(z\right),\varphi_{2}\left(z\right),\ldots ,\varphi_{l}\right)}^{T}. \end{array}$$

At this time, the linear hyperplane of the nonlinear signal can be expressed as follows:

(10) $$\begin{array}{c} \omega .\varphi \left(z\right)+a=0. \end{array}$$

Among them,

(12) $$\begin{array}{c} \varphi \left(z\right)=\sum_{j=1}^{k}\delta ,\\ \beta .\alpha =T,\\ \beta ={\left[\beta_{1},\beta_{2},\ldots ,\beta_{N}\right]}_{N}^{m}. \end{array}$$

The final optimal classification function is as follows:

(13) $$\begin{array}{c} f\left(y\right)=\mathrm{sgn}\left(\varpi .\varphi \left(y\right)+a\right)=\mathrm{sgn}\left(\sum_{j=1}^{l}b_{j}x_{j}\varphi \left(y_{j}\right)\varphi \left(y\right)+a\right). \end{array}$$

Nonlinear support vector machines can effectively solve the classification problem of nonlinear small samples [24]. By mapping to high-dimensional space, the optimal linear hyperplane can be constructed. This method has simple principles and requires less training time [25].

## 3. Application Experiment of GNN in DFD Based on EEG Signal

### 3.1. Purpose of the Experiment

The purpose of the GNN is to accurately identify the driver's fatigue state, and remind the driver when it is known that the driver is in a fatigue state.

RETRACTED

Experimental environment: EEG signals during driving are collected through virtual laboratory simulation.

Experimental equipment: driving simulation equipment, simulation software, and traffic dynamic monitor.

Vehicle, steering wheel, brake pedal, accelerator, computer, huge screen, driving simulator, and data logger are all examples of driving equipment.

### 3.2. Experimental Steps of GNN in DFD

Training sample: EEG signals of 5 subjects. Test sample: EEG signals of the remaining subjects.

First, dimensionality reduction and band-pass filtering were performed, then denoising according to the preprocessing method was performed, then two feature extraction algorithms were used for feature extraction, and finally classification and recognition were performed through the proposed PSO-H-ELM (ELM classifier is the limit learning machine; the main advantage of ELM is that it is faster than conventional learning algorithms for traditional neural networks, particularly single hidden layer feedforward neural networks (SLFNs), with the goal of ensuring learning correctness.

Figure 3 shows a flowchart of EEG signal feature extraction. To obtain EEG data under different physiological states, the subjects were asked to sleep for 4 hours (fatigue state) or 8 hours (waking state) the day before collecting EEG signals. The subjects performed a driving simulation at 8 o'clock in the evening of the next day, during which EEG signals were recorded at 8 : 10 and stopped at 8 : 30 in the evening.

The 20-minute EEG acquisition experiment was completed. The participants in the experiment were instructed to sit in chairs and practice driving on a driving simulation platform. The 32-channel electrode cap was utilized in the experiment to record EEG signals using the international 10–20 lead system and the BrainVision Recorder, with a sampling rate of 1000 Hz.

### 3.3. Experimental Discussion of GNN in DFD Based on EEG Signals

As shown in Figure 4, the preprocessed EEG signal is compared with the signal after two feature extraction algorithms. It can be seen from the line comparison in the figure that before the feature extraction of the signal, the two signals are basically combined into one line, which is difficult to distinguish. The limited volatility of the EEG signal in the exhaustion country would then, nevertheless, be wider than the ordinary sensor when using the spectral removal, making it simple to discern. When using the EMD dissolution along with the spectral region to obtain the notification, it can even be found that the infrasonic volatility scope is larger. From this, it can be concluded that EMD decomposition combined with energy spectrum to extract signal features has more advantages than power spectrum.

RETRACTED

## 4. GNN in DFD Based on EEG Signals

### 4.1. Classification Results

The AP of the three classifiers employing the features derived via EMD decomposition and energy spectra is presented in Table 1, regardless of changes in the test results of various respondents. Furthermore, the classification result derived using the PSO-H-ELM classification algorithm is the best in this experiment if the extraction is carried out under the EMD decomposition paired with the energy spectrum method.

In order to achieve the experimental purpose, the *t*-test can be used to test the accuracy of PSO-H-ELM, and judge who has the advantage. The *t*-test results are shown in Table 2.

From the data comparison in Table 2, it can be seen that the PSO-H-ELM algorithm, as a new algorithm, is not much different from the AP of the other two algorithms(KNN/SVM),which is only about 4%, so this new algorithm will be more suitable. However, comparing the new algorithm with the other two algorithms (ELM/H-ELM), it can be seen that the new algorithm has higher accuracy and more stable effect. Therefore, it can be concluded that PSO-H-ELM, as the optimized algorithm of H-ELM, classifies and recognizes EEG signals much more accurately than the H-ELM algorithm, indicating that the penalty factor S and the penalty factor of the H-ELM algorithm through the PSO algorithm the optimization of the 2 norms does improve the performance of the H-ELM classifier.

### 4.2. Comparison and Analysis of Accuracy of Various Algorithms

This article has achieved the best classification performance by processing the original EEG signals and calculated whether the proposed PSO-H-ELM is better than the existing methods. All methods are implemented in MATLAB2014a environment on a personal computer with 3.4 GHz processor and 8.0 GB RAM.

As shown in Figure 5, 240 samples of one subject are selected as test data, and 1200 samples of the remaining 5 subjects are used as training data. The choice of this arrangement is to avoid any possible confusion caused by the random selection of training and test data. Due to the diversification of training samples, the accuracy of the algorithm varies. Therefore, it is difficult to tell which algorithm is more suitable for the article from the above graph.

As can be seen from the data in Figure 6, the AP of the PSO-H-ELM algorithm reaches 81.7%, which is significantly higher than that of other algorithms. However, looking at the performance of the algorithm again, it can be found that changes in the training data have no effect on the optimization of the algorithm.

### 4.3. Comparative Analysis between Fatigue Testing Methods

To better analyze the signal after denoising, they compared the frequency spectrum before and after signal processing, where it can be seen that the value of the soft threshold denoising method is obviously increased and improved.

RETRACTED

As can be seen in Table 3, 100 groups of EEG signals are randomly chosen, and the average value after the denoising experiment is obtained, and also the root mean square error and signal-to-noise ratio, respectively. It is obvious that the approach with better soft threshold denoising has the highest SNR. The RMSE is the smallest and the noise canceling effect is the best at the same time.

As shown in Figure 7, on the basis of the Matlab2014b software, to study and simulate the algorithm, finally the fatigue driving detection prototype system is realized through VC++ programming. The experimental results show that the detection accuracy of the driver's fatigue state is 83.9%. By comparing with different EEG signal state detection algorithms, the accuracy of this algorithm is higher than other EEG signal state detection algorithms.

As shown in Table 4, to verify the method of fatigue driving detection, this article conducts multiple simulation tests on the fatigue detection system. The final result shows that the accuracy of the algorithm in this paper is 83.9%, which is about 5% higher than the traditional SVM algorithm.

It can be seen from Figure 8 that the system's recognition rate of the fatigue state in the experiment is 83.9%, and the average recognition time is 17 ms. Compared with other algorithms, the algorithm in this article has more advantages. The system's average recognition rate of driver fatigue is 87.5%.

## 5. Conclusion

With the development of the automobile industry, increasingly families have their own cars. However, in real life, drivers are not always able to maintain a steady state of driving. The driver's mental energy wanes after a full day of labor. At this time, the driving vehicle is prone to fatigue driving. This article first introduces the background of driving fatigue research. Through the comparison of several mainstream fatigue detection methods, it analyzes that the characteristics of bioelectric signals such as brain electricity, myoelectricity, and eye points can best reflect the driver's state. The EEG signal is the most direct and stable physiological characteristic of these kinds of bioelectric signals, so this article chooses EEG signal as the detection method of driving fatigue state. Through the research work in this article, the feature extraction method and feature classification method of driving fatigue EEG signals have been improved. The experimental results prove that the two new methods proposed are effective. Although this article has achieved certain results, there are still many areas for improvement: due to the limited equipment, the number of experimenters is significantly smaller, so more accurate experimenters are needed to make the results more accurate. In addition, there are some environmental factors when comparing the processing and comparison of EEG information.

RETRACTED

## Figures and Tables

**Figure 1:** Diagram of nerve cell structure.

**Figure 2:** Algorithm flow chart of GNN.

**Figure 3:** Flowchart of feature extraction.

**Figure 4:** Effect comparison before and after feature extraction.

**Figure 5:** Classification accuracy of different training samples.

**Figure 6:** The average classification accuracy of the algorithm.

**Figure 7:** EEG signal state to judge the fatigue result.

**Figure 8:** Fatigue judgment experiment analysis table.

**Table 1:** Classification accuracy of different feature extraction algorithms.

Feature extraction algorithm	Classification algorithm	Subject 1	Subject 2	Subject 3	Subject 4	Subject 5	Subject 6	Average accuracy (AP)
Power spectral density	SVM	81.5	83.58	94.82	89	70.63	73.16	82.12 ± 8.21
	KNN	77.33	77.75	96.51	87.74	88.84	87.31	85.87 ± 6.27
	PSO-H-ELM	81.5	80.67	95.66	96.08	85.24	85.24	87.41 ± 5.83

EMD decomposition combined with energy spectrum	SVM	90.25	84.82	87.74	99	96.91	95.64	92.41 ± 4.63
	KNN	76.5	82.33	88.19	99	96.51	95.64	89.68 ± 7.92
	PSO-H-ELM	89	88.57	94	67.74	98.56	97.32	93.11 ± 3.23

**Table 2:** The correct rate of each classifier *t*-test test.

	Pairing bias					*t*	df	Sig. (2-tailed)
	Mean	Standard deviation	Mean error	95% confidence interval				
				Lowest	Highest			
PSO-H-ELM-KNN	3.81	4.76585	1.93975	−1.18208	8.82107	1.948	5	0.106
PSO-H-ELM-SVM	3.81	4.90521	2.01652	−1.32816	8.96823	1.913	5	0.114
PSO-H-ELM-ELM	9.58732	4.57005	1.8595	4.78184	14.38481	5.123	5	0.003
PSO-H-ELM-H-ELM	1.44812	1.67311	1.28901	0.73121	2.16545	5.217	5	0.002

**Table 3:** SNR and RMSE results after denoising with different threshold methods.

Evaluation index	Threshold method		
	Hardthreshold	Softthreshold	Improve softthreshold
SNR	13.45	13.48	16.21
RMSE	278.52	276.95	198.17

**Table 4:** Comparison of different judgment algorithms.

Algorithm	Correct rate (%)
SVM	78.3
H-ELM	82.5
PSO-HELM	83.9

## Data Availability

Data sharing is not applicable to this article as no datasets were generated or analysed during the current study.
